The article "Genomic Characteristics of Chinese Borrelia burgdorferi Isolates" was published in 2016. Journal: PLoS One.

# Genomic Characteristics of Chinese *Borrelia burgdorferi* Isolates

**DOI:** 10.1371/journal.pone.0153149

**Published:** 2016-04-19

**Authors:** Qin Hao, Pengcheng Du, Wen Zhang, Xuexia Hou, Lin Zhang, Yuanyuan Zhang, Huixin Liu, Wei Liu, Chen Chen, Kanglin Wan

**Affiliations:** 1 State Key Laboratory of Infectious Disease Prevention and Control, National Institute for Communicable Disease Control and Prevention, Chinese Center for Disease Control and Prevention, Beijing, 102206, China; 2 Collaborative Innovation Center for Diagnosis and Treatment of Infectious Diseases, Hangzhou, 310003, China; University of Kentucky College of Medicine, UNITED STATES

## Abstract

In China, *B*. *burgdorferi*, *B*.*garinii*, *B*. *afzelii* and *B*. *yangtze* sp. nov have been reported; *B*.*garinii* and *B*. *afzelii* are the main pathogenic genotypes. But until now only one Chinese strain was reported with whole genome sequence. In order to further understand the genomic characteristics and diversity of Chinese *Borrelia* strains, 5 isolates from China were sequenced and compared with the whole genome sequences of strains in other areas. The results showed a high degree of conservation within the linear chromosome of Chinese strains, whereas plasmid showed a much larger diversity according to the majority genomic information of plasmids. The genome sequences of the five Chinese strains were compared with the corresponding reference strains, respectively, according to the genospecies. Pairwise analysis demonstrates that there are only 70 SNPs between the genomes of CS4 and B31. However, there are many more SNPs between the genomes of QX-S13 and VS116, PD91 and PBi, FP1 and PKo, R9 and Pko, respectively. Gene comparison showed some important different genes. OspA was one of the important different genes. Comparative genomic studies have found that OspA gene sequences of PD91 and R9 had great differences compared with the sequence of B31. OspA gene sequence of R9 had a 96bp deletion; OspA gene of PD91 had two deletions: 9bp and 10 bp. To conclude, we showed the genomic characteristics of four genotype Chinese *B*. *burgdorferi* strains. The genomic sequence of *B*. *yangtze* sp. nov and differences from *B*. *valaisiana* were first reported. Comparative analysis of Chinese strains with the different *Borrelia* species from other areas will help us to understand evolution and pathogenesis of Chinese *Borrelia burgdorferi* strains.

## Introduction

*Borrelia burgdorferi* sensu lato, which is the agent of Lyme disease, is a genetic diversity complex[1–5]. Up to now at least 15 genospecies have been described: *B*. *burgdorferi* sensu stricto, *B*. *garinii*, *B*. *afzelii*, *B*. *japonica*, *B*. *valaisiana*, *B*. *lusitaniae*, *B*. *andersonii*, *B*. *tanukii*, *B*. *turdi*, *B*. *bissettii*, *B*. *sinica*, *B*. *spielmani*, *B*. *californiensis*, *B*. *yangtze* sp. nov and *B*. *carolinensis* sp. nov[6–10]. In China, more than 100 strains were isolated from ticks, animals and patients[11]. There are five species reported by several studies: *Borrelia burgdorferi*(sensu stricto), *Borrelia garinii*, *Borrelia afzelii*, *Borrelia sinica*, and *Borrelia yangtze* sp. nov[6, 11, 12].

The article "Genomic Characteristics of Chinese Borrelia burgdorferi Isolates" was published in 2016. Journal: PLoS One.

*B*. *yangtze* sp. nov is a group of *B*. *valaisiana*-related strains, which is distributed in eastern Aisa. According to the reports, There are phenotypic differences between *B*. *valaisiana* and *B*. *yangtze* sp. nov[13]. But there are no reports about the genomic differences between them.

To date, whole genome sequences of 26 Lyme disease spirochete strains have been reported: 15 *B*. *burgdorferi isolates*, 3 *B*. *afzelii isolates*, 5 *B*. *garinii* isolates, 1 *B*.*bavariensis* sp. nov. isolate, 1 *B*. *bissettii* isolate, 1 *B*. *valaisiana* isolate, and 1 *B*. *spielmanii* isolate[14–21]. Among all these strains, only 1 strain (*B*. *garinii* NMJW1, isolated from Ixodes persulcatus) comes from China[18].

In order to gain the genomic information of Chinese *B*. *burgdorferi* strains, Five Chinese isolates, including 2 *B*. *afzelii* isolates and 1 isolate of *B*. *burgdorferi* sensu stricto, *B*. *garinii*, and *B*. *yangtze* sp. nov respectively, were sequenced and compared with the whole genome sequences of strains in other areas.

## Materials and Methods

### Strains

Five *B*. *burgdorferi* isolates were chosen for whole genome sequencing analysis: CS4 from *B*.*b*.*s*.*s*, PD91 from *B*. *garinii*, FP1 and R9 from *B*. *afzelii*, QX-S13 from *B*. *yangtze* sp. nov (Table 1).

**Table 1:** Information of 5 isolates.

Strains	Biological source^[^^11^^]^	Region	Genospecies^[^^12^^]^	Passages
CS4	*Caprolagus sinensis bladder*	Hunan	*B*. *burgdorferi* sensu stricto	>30
PD91	Patient blood	Inner Mongolia	*B*. *garinii*	>30
FP1	Patient blood	Sichuan	*B*. *afzelii*	<30
R9	Patient CSF	Heilongjiang	*B*. *afzelii*	<30
QX-S13	*Apodemus agrarius*	Guizhou	*B*. *yangtze* sp. nov	<15

### DNA extraction

DNA was extracted by a modification of a method previously described [12]. After 20 min incubation at 37°C, 80μl of 10% SDS was added to the preparation (10μg in 1ml of PBS), and the preparation was heated at 65°C for 10min. Next, 20μl of RNase (10mg/ml) was added, and the solution was incubated at 37°C for 2h. Following the addition of 10μl of proteinase K, the preparation was incubated at 37°C for 2h. Next, the DNA was extracted two times with equal volumes of phenol and once with an equal volume of chloroform. The DNA was precipitated by adding two volumes of absolute ethanol. The precipitated DNA was washed with 70% ethanol and resuspended in TE (pH 8.0).

The article "Genomic Characteristics of Chinese Borrelia burgdorferi Isolates" was published in 2016. Journal: PLoS One.

### Genome sequencing, assembling and annotation

A genome shotgun method was used to acquire the genome sequence. DNA library of 500-bp fragments was constructed for high throughput genome sequencing with Illumina GAIIx sequencer and pair-end 75-bp reads were collected. We obtained, in total, 127~199 Mb reads for each strain covered 85~133 folds of the reference genome from B31[14]. By mapping to chromosome and plasmids of references, raw reads of each strain were located to chromosomes and plasmids, and then assembled by SOAPdenovo software respectively. The assembled sequences were analyzed by our automatic analysis pipeline, including gene prediction by Glimmer[22], gene annotation by compared to different databases of NT, NR and swissport with BLAST, and gene function prediction based on COG and InterproScan databases. Gene pathways were annotated based on KEGG.

### Comparative genomic analyses

Whole-genome raw SNPs (single nucleotide polymorphisms) were detected by mapping high-throughput SOLEXA read to reference genome using SOAP software with default parameters[23]. Insertions and deletions were detected by comparing the assembled genome with the reference genome using BLAST software.

### Core genome analysis and phylogenetic reconstruction

Orthologous genes were detected by OrthoMCL software version 1.4[24] in 31 *Borrelia burgdorferi* strains including ours. The genes related with lateral gene transfer or recombination event were removed to get core genes. Gene differences were calculated from the distribution of orthologous genes in each genome. Phylogenetic relationship was reconstructed using concatenated amino acid sequence of core genes by Mega software using Neighbor-Joining method.

## Results

### Genomic features of 5 sequenced Chinese isolates

The draft-quality chromosome sequences of the five strains, CS4, FP1, R9, PD91 and QX-S13 were sequenced and assembled into 3, 3, 5, 5 and 5 scaffolds, with N50 are 469678-bp, 463417-bp, 463437-bp, 277204-bp and 467615-bp respectively. Table 2 shows the genomic festures in details.

**Table 2:** Genomic features of 5 sequenced *B*. *burgdorferi* isolates in China.

Genome Feature	CS4	PD91	FP1	R9	QX-S13
G+C content(%)	28.55	28.39	28.28	28.24	28.05
# of ORFs	829	832	828	846	851
% of ORFs in Genome	93.14	92.88	93.25	92.67	92.80
Average Length of ORFs	1019.17	1009.82	1017.47	1004.60	997.88

### Plasmids

Besides the chromosome, the plasmids of five sequenced strains were also be represented at least in part in the shotgun data (coverage>50%). We found that there are varying amounts of plasmids in the genome of the five Chinese strains compared with the B31 strain, including circular plasmids and linear plasmids (Table 3).

The article "Genomic Characteristics of Chinese Borrelia burgdorferi Isolates" was published in 2016. Journal: PLoS One.

**Table 3:** Part of the plasmids of 5 sequenced chinese *B*. *burgdorferi* isolates compared with B31strain.

Strains	Genotype	Circular plasmids	Linear plasmids
B31	*B*.*b s*.*s*	cp9, cp32-1, cp32-3, cp32-4, cp32-6, cp32-7, cp32-8, cp32-9, cp26	lp17, lp25, lp28-1, lp28-2, lp28-3, lp28-4, lp36, lp38, lp54, lp56, lp21, lp5
CS4	*B*.*b s*.*s*	cp9, cp32-1, cp32-3, cp32-4, cp32-6, cp32-7, cp32-8, cp32-9, cp26	lp17, lp28-3, lp54
PD91	*B*.*garinii*	cp9, cp32-1, cp32-3, cp32-4, cp32-6, cp32-7, cp32-8, cp32-9, cp26	Lp17, lp25, lp28-2, lp28-3, lp28-4, lp54, lp56, lp5
FP1	*B*.*afzelii*	cp32-1, cp32-3, cp32-4, cp32-6, cp32-7, cp32-8, cp32-9	Lp17, lp21, lp25, lp28-2, lp28-4, lp54
R9	*B*.*afzelii*	cp9, cp32-1, cp32-3, cp32-4, cp32-6, cp32-7, cp32-8, cp32-9, cp26	Lp17, lp25, lp28-2, lp28-4, lp54
QX-S13	*B*. *yangtze sp*. *nov*		lP54

### Comparative genomic analyses

#### Genome SNPs

The genome sequences of the five Chinese strains were compared with the corresponding reference strains respectively according to the genospecies. Pairwise analysis demonstrates that there are only 70 SNPs between the genomes of CS4 and B31. However, there are much more SNPs between the genomes of QX-S13 and VS116, PD91 and PBi, FP1 and PKo, R9 and Pko respectively (Table 4).

**Table 4:** SNP number of each genotype.

Genotype	Query	Reference	SNPs
*B*. *burgdorferi*	CS4	B31	70
*B*. *garinii*	PD91	PBi	10988
*B*. *yangtze* sp.nov.	QX-S13	VS116	16724
*B*. *afzelii*	FP1	PKo	3804
*B*. *afzelii*	R9	PKo	3686

### Polymorphism of OspA gene

Comparative genomic studies have found that OspA gene sequences of 5 Chinese strains had great differences compared with the sequence of B31. OspA gene sequence of R9 had a 96bp deletion (147–242); OspA gene of PD91 had two deletion: 9bp (647–655) and 10 bp (657–666) (Fig 1).

**Fig 1:** Comparison of ospA gene of 5 chinese strains with B31.

### Phylogenetic tree of Chinese strains and the ones in other areas

The result of phylogenetic analysis of 5 Chinese strains and 26 reference strains based on the whole genome showed all *Borrelia burgdorferi* strains had a same ancestor. The phylogenetic tree identified two pairs of statistically supported sister-group genomes from China: FP1-R9 and PD91-NMJW1(Fig 2).

**Fig 2:** Whole genome phylogenetic analysis of 5 chinese strains and 26 reference strains.

## Discussion

5 strains in this study comes from 4 genotypes in China: CS4 isolated from the bladder of a hare *Caprolagus sinensis* in Hunan province is the reference strain of *B*.*b*.*s*.*s* genospicies. Its whole genome sequence analysis helps to understand the Chinese *B*.*b*.*s*.*s* genetic characteristics and differences from American *B*.*b*.*s*.*s* strains. PD91 was isolated from the blood of a patient suffered from mental abnormality diagnosed clinically in Inner Mongolia, FP1 from the blood of a patient with facial paralysis in Nanchuan county, Chongqing city, R9 from the cerebrospinal fluid of a patient with chronic meningitis in Mudanjiang, Heilongjiang province. Their whole genome sequences help to understand Chinese *B*. *garinii* and *B*. *afzelii* genetic information and differences from the European *B*. *garinii* and *B*. *afzelii* strains respectively; QX-S13 originating from the kidney of *Apodemus agrarius* in Guizhou province, belongs to *B*. *Yangtze sp*. *nov*. Its whole genome sequence can clear *B*. *Yangtze sp*. *nov*. genetic differences from *B*.*valaisiana* strain.

The article "Genomic Characteristics of Chinese Borrelia burgdorferi Isolates" was published in 2016. Journal: PLoS One.

The genome sequences of 5 Chinese *B*. *burgdorferi* strains were compared respectively with the corresponding reference strains according to the genospecies. The results showed that there is the different length of Chromosomes in the different strains. Length differences of Chromosomes in sequenced strains were mainly focus on telomeric regions, which is consistent with the reports[16, 25].

Genome SNPs analysis showed there were much more SNPs between *B*. *Yangtze sp*. *nov*. strain QX-S13 and *B*. *valaisiana* strain VS116 (16724 SNPs), *B*. *garinii* strains PD91 and PBi (10988 SNPs).

Comparative genomic studies have found that OspA gene sequences of 5 Chinese strains had great differences compared with the *ospA* sequence of B31. OspA acts as an adhesin, and is required for spirochetes to successfully colonize in the tick midgut. But when the arthropod engorges on a host, OspA is down-regulated[26]. OspA gene variation shows *B*. *burgdorferi* adapts to diverse environments in the tick and mammal during its life cycle.

Sequence analysis of plasmids showed that the numbers of plasmids in 5 sequenced strains are different. But cp26 and lp54 or their homologous plasmids exist in all 5 strains. According to the reports[15, 16], The core of B.b.sl genomes consists of the chromosome and two plasmids collinear between all species. Additionally, strains can loose some plasmids due to a lack of selection pressure.

Whole genome phylogenetic analysis of 5 Chinese strains together with 26 reference strains identified two pairs of statistically supported sister-group genomes from China: FP1-R9 and PD91-NMJW1. FP1 was isolated from facial paralysis patient’s blood in Nanchuan county, Sichuan province, R9 was isolated from chronic meningitis patient’s cerebrospinal fluid in Mudanjiang, Heilongjiang province. Our investigation results showed that this kind of *B*. *afzelii* strains could cause neurogenic borreliosis and also distributed widely in China. PD91 and NMJW1, which belong to *B*. *garinii*, were isolated from Inner Mongolia. PD91 isolated from the blood of a patient suffered from mental abnormality and NMJW1 from *Ixodes persulcatus* were highly similar sequences, which could provided evidences for the spread of this kind of strains and proving that *Ixodes persulcatus* is a main vector in the transmission of *Borrelia burgdorferi* in Inner Mongolia.

The article "Genomic Characteristics of Chinese Borrelia burgdorferi Isolates" was published in 2016. Journal: PLoS One.

To conclude, we showed the genomic characteristics of four genotype Chinese *B*. *burgdorferi* strains. The genomic sequence of *B*. *yangtze* sp. nov and differences from *B*. *valaisiana* were first reported. Comparative analysis of Chinese strains with the different *Borrelia* species from other areas will help us to understand evolution and pathogenesis of Chinese *Borrelia burgdorferi* strains.
